The article "Music Teaching Management and Music Culture Communication Environment Based on Ergonomics" was retracted in 2023. Reasons: unreliable results or conclusions; concerns about the data; concerns about the results or conclusions; concerns about the peer review.

# Music Teaching Management and Music Culture Communication Environment Based on Ergonomics

**DOI:** 10.1155/2022/4186092

**Published:** 2022-09-14

**Authors:** Rui Dong

**Affiliations:** The Arts Faculty of North University of China, North University of China, Taiyuan, Shanxi 030051, China

## Abstract

Music education has a relationship that is mutually restraining and interdependent. The necessity of spreading music culture offers music education social relevance and existential value in the history of music culture's growth, and the method of spreading music culture—music education—injects strength and life into the development of music culture. Music pedagogy is constrained by the evolution of music culture as a whole. In terms of music pedagogy, traditional culture and their peculiarities or qualities will have an impact on the creation of the curriculum content system, which is also the main topic of music teaching management. By using anthropometry, physiological and psychological measurement, etc. with the human body as the main body, ergonomics is the study of the reasonable coordination between the structure and function of the human body, psychology, mechanics, and music teaching methods in order to satisfy people's physical and mental activities and achieve the best use efficiency. The focus should be on comfort, great performance, safety, and health. In order to create a model for evaluating the quality of music instruction, a back propagation neural network (BPNN) is optimised in this paper using an adaptive mutation genetic algorithm. According to the research, our approach outperforms the BPNN model optimised using conventional evolutionary algorithm by 20.21%. The convergence pace is 80.11% faster than the convergence speed of a conventional genetic algorithm. The comparative result demonstrates that the BPNN teaching quality evaluation model with genetic algorithm optimization based on adaptive mutation can produce a more logical scientific evaluation result for the quality of music instruction.

## 1. Introduction

Music education and music culture are not the same thing. A necessary but not the sole requirement for the emergence and advancement of music culture is music education. We also understand that since music culture is a cultural means of expressing ideas through music, it is inescapably influenced by the national traditional culture and has unique national features [1]. We examine the connection between music education and music culture at the spiritual level of music culture while considering music education to be a component of music culture [2]. However, it must be emphasized that the music education activities and the music theory research in the music culture belong to the system level and the spirit level of the music culture, respectively. Because, music education activities are bound to be closely linked with the dissemination of music culture, school music education must be institutionalized music culture dissemination [3]. Under the background of the rapid development of mass music communication, in order to further improve the effectiveness of teaching, we must consider the impact of music communication on students. This requires that our music teaching must pay attention to social music, so that students' interpretation of social music presents a consistent music learning concept [4]. Combined with the application of ergonomics, its basic data has three aspects: human body scale, human body structure, and human body action domain. These aspects will be used in music teaching. Among them, one of the basic data of ergonomics research is the human body scale. It is of profound significance to strengthen the research on human body scale in music teaching methods to ensure the practicality of teaching programs [5].

The article "Music Teaching Management and Music Culture Communication Environment Based on Ergonomics" was retracted in 2023. Reasons: unreliable results or conclusions; concerns about the data; concerns about the results or conclusions; concerns about the peer review.

Music education is the manifestation of music culture dissemination and an important part of music culture dissemination. For music theory research that belongs to the spiritual level of music culture dissemination, it shoulders the responsibility of disseminating research results through music education, providing benefits, and creating value for the entire music culture dissemination, music academic field, and even the entire society [6]. The tradition of music culture dissemination restricts the process of music education. Different music education reflects different backgrounds of music culture dissemination and presents different music culture dissemination traditions and national spirits [7]. After a systematic analysis of each link in the music teaching evaluation system, it is not difficult to see that there are many undetermined factors in the teaching evaluation system. The main reason is that there are certain human subjective factors in the evaluation results and data analysis process. The results of teaching quality evaluation have errors and do not have universal applicability [8]. As can be observed, dealing with the assessment process' mistake sources is the crucial first step in improving the teaching evaluation system. The experimental environment for model testing and training as well as the collection of experimental data are built in this study. The data are preprocessed in accordance with the specifications of the input vector of the model for evaluating the quality of instruction. Second, the determination of parameters in the genetic algorithm and BPNN in the teaching quality evaluation model is explained in accordance with the starting parameter value established by empirical formula and ongoing experiments.

The article "Music Teaching Management and Music Culture Communication Environment Based on Ergonomics" was retracted in 2023. Reasons: unreliable results or conclusions; concerns about the data; concerns about the results or conclusions; concerns about the peer review.

Music culture carries the culture of the entire region, so local music is closely related to the national culture of the country. Only by maintaining this mutually beneficial and win-win relationship can the national culture be further developed [9]. In the context of multicultural dissemination, the limitation of traditional teaching thinking should be broken, and cultural factors should influence and promote educational reform. The most realistic curriculum setting method to implement the principle of pluralism in the current higher music education activities is to integrate the cultural essence and characteristics of various ethnic groups in the world into the existing curriculum. On the basis of the current higher music education courses, integrating the essence and characteristics of the music culture of various nationalities in the world can not only broaden students' horizons, but also enable students to contact more music culture forms and skills, so that students can experience the characteristics of the music of various nationalities in the world and the essence of music culture in the music teaching courses, and on this basis, carry out the refining, development and innovation of music art [10]. The people-oriented principle must constantly guide the implementation of ergonomics in music education. The two main manifestations of the application of ergonomics in music education are the spiritual function and the practical function. Indoor environments have an impact on people's psychological environments, and effective music instruction can assist students' mental health to some level [11]. Contrarily, the primary goal of a music teaching strategy is to satisfy the needs of the students; therefore, design must take into account the teaching strategy's practicality. These are the benefits of this research:

1. A neural network-based teaching quality evaluation model is built on the basis of examining the benefits and drawbacks of the earlier teaching quality evaluation methods and summarising the current teaching quality evaluation model methods, aiming to address the limitations of the existing evaluation methods
2. Comprehensive management of provided teachers, students, and system information through database technology and network technology. Compared with manual processing, computer management data is more accurate, and data processing is faster, which creates conditions for the realization of systematic management of evaluation information and automatic statistical data, reduces the workload of teaching evaluation work, and shortens the time for evaluation implementation

The article "Music Teaching Management and Music Culture Communication Environment Based on Ergonomics" was retracted in 2023. Reasons: unreliable results or conclusions; concerns about the data; concerns about the results or conclusions; concerns about the peer review.

## 2. Related Work

Li believes that in the process of music culture dissemination, the inheritance and dissemination of the artistic characteristics of national music also needs the artistic characteristics of national music to form its own style and stage. In the current development, the stereotyped pop music is too monotonous due to the lack of fresh elements for a long time, and its form is too uniform, which is not conducive to people forming emotional resonance [12]. Xia explored the relationship between the current music teaching reform and music culture dissemination in universities and hoped that through such efforts, it would play a role of throwing bricks and attracting jade, make the clues of relevant issues more clear, and form a benign interaction between the music teaching reform in colleges and universities and the social music culture dissemination, to promote common development [13]. Blackburn proposed in his book that with the upgrading of equipment and technology, the production cycle of music works is greatly shortened, and the cost and threshold of communication are greatly reduced. The convenient age of integrated media has brought more opportunities for the dissemination of music culture and further stimulated people's desire for music creation [14]. Ruijun believes that in order to truly realize the diversification of music teaching, it is necessary to bring the music culture of various nationalities into the classroom. Through classroom teaching, students can understand the music culture characteristics of various nationalities, absorb the essence of them, and expand their horizons [15]. Huang pointed out that it is necessary to design and arrange music teaching courses reasonably, link diversified music culture with music teaching, so that students can understand and learn more thoroughly, and then integrate them [16]. Yang has deeply studied the ways and means of implementing diversified music teaching and discussed the requirements for teachers and the future development prospects of the implementation of diversified music teaching functions, which also makes the teaching contents, methods, objectives, and even teaching concepts of music teaching more diversified and scientific [17]. Chang was inspired by the concept of ergonomics and studied the design of multimedia courseware that better meets the physical and psychological needs of teachers and students [18]. Michelle proposed to introduce the theory of artificial neural network into the teaching quality evaluation system, which not only solved the problem of qualitative and quantitative indicators in the comprehensive evaluation index system but also avoided the direct influence of human factors on the evaluation results. To make the evaluation more accurate and effective, the teaching quality evaluation model established by neural network theory is an effective method for teaching quality evaluation [19]. Huang assumes that our design conforms to the characteristics of human brain physiology and psychology, and the learning efficiency of learners will be greatly improved [20]. Therefore, all the work of courseware design must be based on evidence. The structure of the courseware, the capacity of the unit, the matching of sound and picture, etc., must conform to the cognitive process and cognitive laws of the brain and psychology. Hao pointed out that the influence of music communication on students is to make people relax, relieve people's mental fatigue, and express people's inner mental pressure. From this, it seems that for the dissemination of mass music, we should grasp and accept it with an appropriate size and a correct attitude [21].

The article "Music Teaching Management and Music Culture Communication Environment Based on Ergonomics" was retracted in 2023. Reasons: unreliable results or conclusions; concerns about the data; concerns about the results or conclusions; concerns about the peer review.

## 3. Interaction between Music Teaching and Music Culture Dissemination

Compared with the music art itself, the music culture mainly relies on communication to develop and inherit. For thousands of years, the spread of music culture has experienced the development and changes from oral communication, cultural transmission to electronic media. Communication allows music culture to flow across time and space, and music culture is constantly changing in the process of communication. The spread of music culture usually includes the music itself, and the ideas are integrated into the works and reflected through the music works. As far as the current higher education curriculum teaching reform is concerned, its basic value pursuit and reform direction are basically the same as that of basic education, emphasizing teaching interaction and paying attention to the comprehensive and balanced development of students. That is, from the perspective of teaching materials, one of the characteristics of the music learning content in the music communication environment is that the learning content is closely related to the learners, or the communication content is closely related to the audience. The closer the content is, the higher the efficiency will be when learning, and the greater the impact on students will be, and the more effective the first definition can be met. As for the teaching content of music teaching, the establishment of school-based music courses in basic education and the development of local music culture resources have high learning effectiveness, as shown in Figure 1.

The article "Music Teaching Management and Music Culture Communication Environment Based on Ergonomics" was retracted in 2023. Reasons: unreliable results or conclusions; concerns about the data; concerns about the results or conclusions; concerns about the peer review.

In the process of music management, all kinds of teaching methods, teaching modes, and functions are changing with each passing day, which need to be maintained and upgraded irregularly. Therefore, the auxiliary teaching system must be expandable and configurable. Music teaching assistant management is implemented by modularization, which can improve the reusability and maintainability of the code by reducing the association between different modules. The design of music assistant management system adopts three-tier architecture, and the specific architecture is shown in the following Figure 2.

This auxiliary music education management system, which is a type of comprehensive education auxiliary management system, is primarily based on the school's music education practises and popular J2EE framework technology to achieve online music education partial auxiliary business office management. It is capable of addressing the needs of both music teachers and students in terms of real-time learning and communication. System testing enables the system to satisfy the demands of financiers and related departments while improving the operating system's efficiency and stability. Friendly user interfaces, comprehensive informational hints, and all manner of friendly errors can direct users to the proper procedure and help them get started right away.

## 4. Teaching Quality Evaluation Model Based on Improved Genetic Algorithm and BPNN

Establishing a more credible and scientific model for evaluating teaching quality is one of the goals of this essay. This model is crucial in advancing teaching quality evaluation. Using the evaluation of the teaching quality of theoretical courses at a university as an example, the information is gathered using a questionnaire in accordance with the system's guidelines. The entropy approach is used to obtain the initial evaluation findings after the data have been preprocessed. The BPNN is then optimised using the modified genetic algorithm to create the teaching quality evaluation model. The model actually consists of two parts. The initial weight and threshold of a BPNN are optimised using an adaptive mutation genetic algorithm in one module, and network training is accomplished using a BP algorithm in the other. A reasonably developed model for evaluating the quality of instruction can be created by combining the two components.

The input layer, hidden layer, and output layer make up the three layers of the feedforward hierarchical network known as the BPNN. The output layer includes:

(1) $$\begin{array}{c} F_{k}=f\left({\text{net}}_{k}\right),\;k=1,2,\cdots ,r,\\ {\text{net}}_{k}=\overset{n}{\underset{i=1}{\sum }}w_{ij}y_{j},\;k=1,2,\cdots ,r. \end{array}$$

Using the gradient descent method to calculate the weight change and the back propagation of the error, the weight change of the output layer is the weight from the *i*th input to the *k*th output:

(2) $$\begin{array}{c} \Delta w_{ki}=-\xi \frac{\partial E}{\partial {w_{ki}}^{2}}=-\xi \frac{\partial E}{\partial a_{k}}\times \frac{\partial a_{k}}{\partial {w_{ki}}^{2}}, \end{array}$$

where the expression of *δ*_*k*_, *e*_*k*_ is:

(3) $$\begin{array}{c} \delta_{ki}=\left(t_{k}-a_{2k}\right)f\left(x_{i}\right)=e_{k}f\left(x_{2i}\right),\\ e_{k}=t_{k}-a_{2k}. \end{array}$$

The network's ability to achieve convergence often dictates how many neurons are placed in the hidden layer. The hidden layer may not be able to be trained or the network may not be “strong” enough to recognise samples that have never been seen before, and the fault tolerance may be inadequate. This is due to the hidden layer having a minimal number of neurons. Using a few empirical formulas, it is possible to estimate the number of neurons in the hidden layer:

(4) $$\begin{array}{c} s=\sqrt{0.41mn+0.11m^{2}+2.34n+0.74m+0.56}n^{2}, \end{array}$$

or

(5) $$\begin{array}{c} s=\sqrt{m+n}+a, \end{array}$$

where *a* is a constant between 1 and 10, *n* is the number of neurons in the input layer, and *m* is the number of neurons in the output layer.

The article "Music Teaching Management and Music Culture Communication Environment Based on Ergonomics" was retracted in 2023. Reasons: unreliable results or conclusions; concerns about the data; concerns about the results or conclusions; concerns about the peer review.

Due to the differentiability of the sigmoid function, the simple differential formula, and easy representation, and its good nonlinear mapping ability, it is mostly used as a mapping function. In this paper, the excitation function of the neurons of the BPNN adopts the sigmoidal function:

(6) $$\begin{array}{c} f\left(x\right)=\frac{1}{1+\exp\left(x_{i}y_{j}\right)/\omega_{ij}}. \end{array}$$

In the process of designing a neural network, the neural network must pass through several different learning rates for training, by observing each training total square error rate of decline to determine whether to choose the appropriate learning rate. If the sum of the squares of the error decreases rapidly, then the learning rate is correct. If the sum-square error shows fluctuation, it indicates that the learning rate is too large.

Get the preliminary evaluation findings by using the entropy approach to calculate the normalised data. The following are the steps involved in the entropy method's calculation:

1. Standardization of the original teaching quality evaluation data, the formula is:

(7) $$\begin{array}{c} {x_{ij}}^{\prime }=\frac{\left(x_{ij}-\bar{x}\right)}{s_{j}} \end{array}$$

In the formula, *x*_*ij*_ is the score value of the *i*th sample in the *j*th index. *x*_*ij*_′ is the standardized value, $\bar{x}$ and *s*_*j*_ are the mean and standard deviation of the *j*th index, respectively. In order to meet the logarithmic requirements in the entropy method, the standardized values need to be shifted:

(8) $$\begin{array}{c} Z_{ij}=x_{ij}+L. \end{array}$$

In the formula, *Z*_*ij*_ is the value after translation, and *L* is the length of translation.

(2) The same quantification of the teaching quality evaluation index, the formula is:

(9) $$\begin{array}{c} p_{ij}=Z_{ij}\overset{n}{\underset{i=1}{\sum }}\bar{Z_{ij}} \end{array}$$

In the formula, *Z*_*ij*_ is the translated teaching quality evaluation data.

(3) Calculate the teaching quality *Q*_*i*_ of the *i*th sample:

(10) $$\begin{array}{c} Q_{i}=\overset{n}{\underset{j=1}{\sum }}\omega_{j}p_{ij} \end{array}$$

In the formula, *ω*_*j*_ is the weight of the *j*th index, *p*_*ij*_ is the *j*th index, and the *i*th sample accounts for the proportion of the index.

The article "Music Teaching Management and Music Culture Communication Environment Based on Ergonomics" was retracted in 2023. Reasons: unreliable results or conclusions; concerns about the data; concerns about the results or conclusions; concerns about the peer review.

## 5. Testing and Analysis

The following list of input techniques will be taught to the BP neural network: the input mode is first transmitted from the input layer to the hidden unit layer, and then, following the processing unit hidden layer, it is sent to the output layer. The results are then compared to the expected values; if the results fall short of the expected values, the error is converted to error-back propagation, which causes the error to travel back along its original path. By adjusting the linking weights of each layer of neurons, the signal error is reduced. This style of alternate forward and backward propagation is referred to as a “memory training” method. The system keeps generalising these two processes through repetition learning, and it will not stop learning when the output value and the predicted value of errors are both within a certain range's upper bound. As soon as a fresh sample is fed into a well-trained network, the corresponding output value can be obtained.

According to the system requirements, database requirements, and the requirements of input items, the test can be placed on the following points: whether the function is realized, whether the data is stored and read correctly, whether the required items are checked, whether the system gives clear prompt information, and whether the page jump is correct when the user triggers the restriction conditions. From the theoretical study, taking the database of the teaching quality part as a comparison object, the system parameters are tested by SPSS software, and the results are shown in Table 1.

Apply the dynamic data management method in the database to the organization of the knowledge base, so that the knowledge base has better operability and maintainability and facilitates the use of functions such as supplement, correction, deletion, and access. At the same time, the complexity of the system design structure is reduced, and it also brings convenience to the related work of system maintenance. Through the verification and testing of the model, we find that it has a positive impact on the evaluation of teaching quality. The results are shown in Table 2.

The article "Music Teaching Management and Music Culture Communication Environment Based on Ergonomics" was retracted in 2023. Reasons: unreliable results or conclusions; concerns about the data; concerns about the results or conclusions; concerns about the peer review.

The subjectivity is very significant when it comes to the content of indicators at all levels of the system for evaluating the quality of teaching because it is frequently decided by the expertise of experts. Since the index system's content cannot be based on subjective opinion, the evaluation's findings are unreliable and should only be used as a guide. The system administrator, who also allows the teachers' permission to download, modify, and maintain pertinent content, is primarily responsible for adding pertinent materials. In parallel, the module automatically records students' browsing based on how often they browse, allowing teachers to assess pertinent popular knowledge. The appropriate teachers publish the music video course materials, and the appropriate permissions are specified. The courseware is accessible to students with the necessary permissions. The system continuously assesses the learning capacity of the students. The system will automatically assess a learner's aptitude for learning and save pertinent data each time they submit their learning outcomes. The revised curriculum is advised to be used in accordance with student difficulty. The following comparisons are made between the suggested course difficulty elements and learner abilities, as shown in Figure 3.

The music teaching auxiliary management system has played a role in promoting the learning of students' music knowledge, the improvement of teachers' work efficiency, and the convenience of leaders' office. The system uses computer technology and network technology, integrates the modern music teaching process, provides rich teaching and learning methods, and facilitates resource sharing and communication. It also can provide some official document auxiliary management functions for school leaders to improve office efficiency. The system requirement analysis phase can use the use case diagram to describe the user requirements of various participants, and the use case diagram can show the participants and use cases of the system, as well as the relationship between them. The purpose of a use case diagram is to model systems and classes, as shown in Figure 4.

When students use the system, they should first submit a registration application to the system, fill in the personal information form, and wait for the system administrator to review after submitting the personal information form successfully. The system administrator will check the student information in the educational administration system according to the various information provided by the students. If the information is correct, the student will be granted the permission to use the system, and then, an email will be sent to the student. Students can then access the system with the username and password they entered when they applied. After logging in to the system, you can view various information announcements, teacher introductions, course introductions, and other information, and then, you can choose courses according to your interests and hobbies. These series of behaviors become the source of data collected by the system and finally form a student feedback information module (Figure 5). The test of this module can verify the effectiveness of the system.

The article "Music Teaching Management and Music Culture Communication Environment Based on Ergonomics" was retracted in 2023. Reasons: unreliable results or conclusions; concerns about the data; concerns about the results or conclusions; concerns about the peer review.

The above introduces the data preparation, mainly including the design of a quantitative questionnaire, the rationality of the questionnaire and the accuracy of the data are tested through reliability analysis and validity analysis, and the questionnaire is distributed and the data are collected, and then preprocess the data involved in the experiment. Then, we need to explain the self-adaptive mutation genetic algorithm and BPNN topology and parameter initialization settings, and apply them to the teaching quality evaluation model to analyze their effects.

The amount of information in the teaching evaluation database has rapidly expanded as online teaching assessment has become more common in the digital campus. Traditional data analysis techniques struggle to extract deep-level meaningful information from the “mountain of” data sets, which can only be accessed via the surface information. An essential goal of teaching evaluation is how to improve the utility of evaluation data to extract information. The accuracy and public trustworthiness of the evaluation results will undoubtedly change, in particular due to the scientific index establishment and rational index weight distribution. Therefore, we compared the traditional BPNN and the improved genetic algorithm to optimize the application of BPNN in the teaching evaluation system, and obtained the results in Figures 6 and 7.

Each neuron in a neural network has the capacity to independently receive, process, and output information; consequently, neurons in the same layer can compute information in parallel and output the results to the following layer of the network for additional processing, allowing the network to operate in real time. The BP neural network is integrated with the entropy approach and genetically optimised using adaptive mutation probability. The algorithm no longer uses gradient descent as its primary optimization method; instead, it simplifies the complex nonlinear optimization problem into an algebraic equation group solution problem, allowing it to quickly determine the weight's global optimum without the need for iterative calculations. It is a polynomial order method with quick calculation times, making it more useful than the BP algorithm.

The article "Music Teaching Management and Music Culture Communication Environment Based on Ergonomics" was retracted in 2023. Reasons: unreliable results or conclusions; concerns about the data; concerns about the results or conclusions; concerns about the peer review.

It is evident that the revised genetic algorithm-based BP evaluation model can produce a rapid, accurate, and scientific evaluation of the teaching quality. The resulting model for evaluating teaching quality has improved convergence and prediction accuracy. In conclusion, the test results demonstrate that the approach utilised in this study outperforms the BPNN model optimised by the conventional genetic algorithm by 20.21%. The convergence speed is 80.11% faster than the genetic algorithm optimization neural network model.

In summary, the test results show that the method used in this paper is 20.21% higher than the BPNN model optimized by the traditional genetic algorithm. In terms of convergence speed, the convergence speed is 80.11% higher than that of genetic algorithm optimization neural network model.

## 6. Music Teaching Development and Cultural Communication Strategy Analysis

As far as music pedagogy is concerned, it is necessary to start from the perspective of pluralism, and only by adopting the perspective of relevance can we make a correct educational judgment. The communicators of music culture should seize the great advantages of new technology in the new era, excavate the value of music culture, promote high-quality music culture, constantly enrich people's cultural and entertainment life by using the integrated media platform and technology, strive to spread music culture to all parts of the world, and make it stand in the forest of music in the world for a long time. Therefore, the author believes that we should start from the following aspects:

1. The selection of music teaching materials shall be based on different schools. For music schools, music teaching materials shall be representative, cover different music cultures, and carefully analyze music theory knowledge, musical instruments, scales, and laws. For comprehensive colleges and universities, it is necessary to choose textbooks that are easy to appreciate and have weak professional knowledge as key teaching materials
2. Music teaching should not only stay at the theoretical stage, but also practice more. We should carry out international music festivals for college students, music sharing meetings for musicians from all over the world, and learn from each other
3. Combined with the application of new media technology, the effect of music communication is further quantified, and the effect of music communication has been further quantified. The communication strategy of music culture needs to strengthen the understanding of the new media era, so as to strengthen the effect of music culture communication and the influence of communication culture in the new media era, transmit the unique music and culture from domestic to international, and give more value and influence to music culture, through communication and inheritance, continuous innovation, and further dissemination

The article "Music Teaching Management and Music Culture Communication Environment Based on Ergonomics" was retracted in 2023. Reasons: unreliable results or conclusions; concerns about the data; concerns about the results or conclusions; concerns about the peer review.

## 7. Conclusions

A genre of art that relies on hearing is music, which is primarily represented in musical compositions and the performance of musical compositions. The field of music culture is directly linked to society, superstructures, and ideas like musicians, musical expertise, and musical aesthetics. Music education is a vital component of music culture, is essential to music culture, and is constantly constrained by music culture as a whole. Music education needs to give more attention to the cause of music education as an essential component of students' intellectual growth. Additionally, it must continually improve music instruction techniques and methodologies while overcoming obstacles. In order to enhance the music teaching activities and the quality of music instruction, carefully compile, sort, and analyse the current music teaching scenario using effective technical tools. It will be easier to learn from and draw on the successful experience of other music culture traditions and music education systems if we examine the relationship between music culture and music education and understand the role of music education in the development of national spirit, the preservation of music culture tradition, the innovation and development of music culture, and its status and role in the inheritance and operation of music culture. The inclusion of foreign music culture in our music education while learning and passing down our own traditional music culture, as well as integrating music learning with a rich national music culture into national music basic education, is currently a crucial endeavour.

## Figures and Tables

**Figure 1:** Music teaching process.

**Figure 2:** The structure of the music teaching assistant management system.

**Figure 3:** Music courseware recommendation effect evaluation diagram.

**Figure 4:** Students participating in the evaluation module test.

**Figure 5:** Student feedback information module test.

The article "Music Teaching Management and Music Culture Communication Environment Based on Ergonomics" was retracted in 2023. Reasons: unreliable results or conclusions; concerns about the data; concerns about the results or conclusions; concerns about the peer review.

**Figure 6:** Improved genetic algorithm to optimize the error sum of squares of BPNN.

**Figure 7:** Improved genetic algorithm to optimize the fitness of BPNN.

**Table 1:** System parameter table structure.

Serial number	Field name	Type	Length	Null	Primary key
1	Registstatue	Integer	1	–	No
2	Loginstatue	Integer	1	–	No
3	Username	Character type	10	–	Yes

**Table 2:** Structure of student score sheet.

Serial number	Field name	Type	Length	Null	Primary key
1	Institutename	Character type	10	–	No
2	Majorname	Character type	10		No
3	Classname	Character type	13	Yes	No
4	Student ID	Character type	17	Yes	No
5	Username	Character type	15	Yes	Yes
6	Passwd	Character type	12		Yes
7	Done	Character type	16		Yes
8	Score	Floating point	11		Yes
9	Grade	Floating point	20		No
10	Question	Integer	6		No

## Data Availability

The data used to support the findings of this study are available from the corresponding author upon request.

## References

[1] Wang R. (2017). J2EE-framework-based development of music assisted teaching management system in universities. *Revista de la Facultad de Ingenieria*.

[2] Sudu L. (2022). Design and application of vocal music teaching management system. *Mathematical Problems in Engineering*.

[3] Zhang C. Y., Amp C. L., University B N (2020). Cross-cultural dissemination of the beauty and connotation of traditional Chinese music culture. *Social Sciences of Beijing*.

[4] Wang J. (2020). Cross-cultural communication discussion on primary school music teaching: how to increase students enthusiasm for learning music. *Music Teaching Research*.

[5] Barton G. (2021). The influence of culture on music teaching and learning. *Australian Association for Research in Music Education*.

[6] Shen W. (2019). Across-culture communication culture teaching. *Journal of Keshan Junior Teachers College*.

[7] Zheng J. (2017). On the role of modern media technology in music communication. *Discussion on the Dissemination of Music Culture*.

[8] Barton G. (2018). The influence of culture on instrumental music teaching: a participant-observation case study of Karnatic and Queensland instrumental music teachers in context. *Contemporary Education and Culture*.

[9] Bing X. U., Jing S. U. (2021). Studies to Chinese college music education management reform and development of countermeasures. *Studies in Sociology of Science*.

[10] Sun G., Fu W. (2021). *E-Learning, E-Education, and Online Training: 6th EAI International Conference, ELEOT 2020, Changsha, China, June 20-21, 2020, Proceedings, Part II*.

[11] Yu R. (2018). The role of musical and cultural factors in music teaching. *Journal of Educational Management*.

[12] Li L. (2018). Research on music teaching mode against the backdrop of "Internet+". *International Management*.

The article "Music Teaching Management and Music Culture Communication Environment Based on Ergonomics" was retracted in 2023. Reasons: unreliable results or conclusions; concerns about the data; concerns about the results or conclusions; concerns about the peer review.

[13] Xia L. Y., University H N (2017). Research on the dissemination and development of the national traditional music culture. *Guizhou Ethnic Studies*.

[14] Blackburn A. (2021). Sourcing gesture and meaning from a music score: communicating techniques in music teaching. *Journal of Research Policy & Practice of Teachers & Teacher Education*.

[15] Ruijun S. U. (2017). Application analysis of interactive teaching model in music classroom teaching of junior middle school. *The Theory and Practice of Innovation and Entrepreneurship*.

[16] Huang M., Arts S. O., University W A (2017). The research of disadvantages of traditional music teaching model in applied undergraduate colleges–Anhui Province as an example. *Journal of West Anhui University*.

[17] Yang Q. (2017). Cloud music teaching database based on opencl design and neural network - science direct. *Microprocessors and Microsystems*.

[18] Chang Y.-J. (2018). A study on the ICT-based traditional music teaching-learning model-focusing on the first grade middle school students. *Journal of Music Education Science*.

[19] Robertson M. M. (2017). Office ergonomics training: an instructional systems model for developing an effective program. *Professional Safety*.

[20] Huang W. W. (2018). Discussion on incoming standard of ISO9000 of teaching quality management in music institutes and departments. *Journal of Fujian Institute of Education*.

[21] Hao Y. (2019). Design and implementation of college music education teaching management system. *Music & Performance*.

